The article "Innovation of Platform Economy Business Model Driven by BP Neural Network and Artificial Intelligence Technology" was retracted in 2023. Reasons: unreliable results or conclusions; concerns about the data; concerns about the peer review; concerns about the citations.

# Innovation of Platform Economy Business Model Driven by BP Neural Network and Artificial Intelligence Technology

**DOI:** 10.1155/2022/3467773

**Published:** 2022-07-09

**Authors:** Lianjie Zhou, Chengfu Wang

**Affiliations:** ^1^Entrepreneurship College, Zhejiang University of Finance & Economics Dongfang College, Haining, Zhejiang 314408, China; ^2^Seoul School of Integrated Sciences & Technologies, Seoul 03767, Republic of Korea; ^3^Information Institute, Zhejiang University of Finance & Economics Dongfang College, Haining, Zhejiang 314408, China

## Abstract

In order to enhance the competitiveness of enterprises, how to evaluate and enhance the competitiveness of B2B e-commerce enterprises and promote the orderly and healthy development of B2B e-commerce industry are discussed. This paper puts forward the research on the innovation of platform economic business model driven by BP neural network and artificial intelligence technology. BP neural network is used to study and evaluate the competitiveness of B2B e-commerce companies. According to the B2B e-commerce company competitiveness theory and BP neural network algorithm, combined with BP neural network and B2B e-commerce company competitiveness evaluation index system, a BP neural network model is designed to analyze the competitiveness of B2B e-commerce enterprises. Determine the expected value of network samples, select *G*1 method to determine the subjective weight, and select entropy weight method to determine the objective weight. With the help of the function in the MATLAB neural network toolbox, the neural network is trained. The results show that when the training times reach 3297 times, the sample mean square error is 9.9869*e* − 06, and the training network reaches convergence. The samples of three enterprises test the trained neural network and input the data of three test samples into the trained BP neural network, and the output results are 0.1531, 0.1371, and 0.1557, respectively. The network model constructed in this paper is effectively close to the training samples. The established BP neural network has good performance and can be used to evaluate the competitiveness of B2B e-commerce companies. Accelerate technological change and realize innovation. Technological capability is the inexhaustible driving force for the development of enterprises. Only with the innovation of keeping pace with the times can application-oriented e-commerce enterprises meet the needs of customers and the market, form the difference between goods or services, and then enable enterprises to win more customers and market share.

## 1. Introduction

Under the background of “Internet Plus,” more and more new ventures choose the platform economic mode as the entry point of innovation in the world. These enterprises have made important contributions to the development of new technologies and the integration of the global economy by constantly subverting and reconstructing the old business models. For example, Taobao, China's largest online shopping retail platform, which creates sales myth every year, does not need to produce any products by itself; Uber, which provides smart travel services worldwide, does not need to provide its own drivers and vehicles; The online takeout trading platform “hungry,” which covers more than 2000 cities in China, does not have its own restaurants and chefs [1, 2]. Under the trend of global economic adjustment, these platform enterprises challenge the traditional enterprise business model with the help of mobile Internet technology and point out a new way for the traditional industry while creating huge profits. Since the government put forward the development strategy of “mass entrepreneurship and innovation,” Internet platform enterprises have always played the role of stormtroopers. Various mass entrepreneurship space platforms provide entrepreneurs with rich entrepreneurial resources, lead start-ups to make changes to the traditional industry pattern, and strive to make enterprises grow into global leaders in the industry [3]. As platform enterprises have created more and more industrial myths, platform, as a leading organizational form in the Internet information age after factories and companies, has been recognized by the industry [3]. As a mainstream business model, the creative destruction nature of platform economy has changed the original business logic. This model can not only bring “win-win” to economic participants, but also realize the value creation of the platform itself. At the same time, there is a rare phenomenon that winners in market competition realize winner take all. As the organizational carrier and value focus of platform economic development, platform enterprises aim to create a unique business ecosystem [4]. This system provides value realization channels for transaction subjects from different types of bilateral markets and promotes the value exchange and interaction of bilateral users.  Figure 1 business model innovation process integration model.

## 2. Literature Review

In response to this research problem, Chen and Ma [5] found that the biggest difference between platform enterprises and traditional enterprises is that the platform does not involve specific transactions; that is, platform enterprises do not produce any specific products for trading subjects. The core task of platform enterprises is to establish a fair and transparent trading platform for buyers and sellers, escort both parties with reasonable and sound trading rules, continuously attract more bilateral users to participate in the platform through unique services, and finally realize the value integration and innovation of the whole trading network [5]. Raddadi and Fava [6] and others believe that compared with traditional unilateral enterprises, platform enterprises have typical characteristics, such as serving bilateral customers, nonneutral price, different roles, and different value orientations. In terms of value creation, as a specific part of a production process, unilateral enterprises can only think about how to create more value from the perspective of the enterprise itself [6]. Thibaut et al. [7] regard platform enterprises as modules based on business ecosystem, and enterprises can provide users with complementary products or services through the platform. At the same time, they believe that we should pay attention to distinguishing between industrial platform and product platform because their building module combination methods are different [7]. On this basis, Fan et al. [8] focused on the differences between industrial platforms and product platforms and proposed that the realization of user value of industrial platforms is mainly through the provision of complementary products and services, which come from different enterprises with complementarity. These enterprises realize complementarity through the technical platform with common reuse basis provided by industrial platforms [8]. Susilo and Liu [9], based on combing the research on platform enterprises at home and abroad, believe that platform enterprises, as the central system in the platform business system, provide an open and connected transaction channel for buyers and sellers with reasonable transaction rules, as a third-party economy providing transaction channels and transaction management. Platform enterprises collect access fees from bilateral users in the market by continuously improving the transaction experience and benefit from successful transactions between buyers and sellers [9]. According to the characteristics of bilateral markets, Yang [10] believes that platform enterprises have the following characteristics: unique value, multicustomer, openness, and complexity and put forward that the platform in “platform enterprises“ can be tangible or intangible. In essence, platform enterprises provide an intermediate layer of transaction (place, media, space, etc.). The middle tier can promote its various groups to reach transactions relatively efficiently and ideally [10]. Tian et al. [11] put forward the classic business model canvas, which is composed of nine elements: customer segmentation, value proposition, sales channel, customer relationship, revenue source, core resources, key business, partners, and transaction structure, which are closely connected and interact [11]. Pierre and Dillenbourg [12] believe that the business model consists of four chain elements that jointly create and deliver value, namely, customer value proposition, profit formula, key resources, and key process [12]. From the perspective of organization, He [13] decomposed the business model into transaction content, transaction governance, and transaction structure [13]. Based on the current research, listed B2B e-commerce enterprises are taken as the research object, an evaluation index system is constructed for its competitiveness, and analysis and research are carried out from four aspects: evaluation index screening, index weight calculation, sample research analysis, and suggestions. BP neural network is selected to train the selected samples to achieve an ideal simulation effect, and the simulation output results are used to evaluate the competitiveness of B2B e-commerce enterprises. It is feasible to evaluate the competitiveness of B2B e-commerce enterprises with the help of BP neural network, and the correct evaluation effect can be obtained; this method also has certain adaptability in evaluating the competitiveness of enterprises in other industries.

## 3. Method

BP neural network is applied to the competitiveness evaluation index system of e-commerce companies.

### 3.1. B2B Selection Principles of Competitiveness Evaluation Indicators of e-Commerce Enterprises

The selected evaluation indicators can not only systematically show the competitiveness of B2B e-commerce enterprises, but also compare the evaluation indicators to identify their weaknesses so as to put forward corresponding improvement suggestions for enhancing the competitiveness of B2B e-commerce enterprises [14]. There are many kinds of evaluation indicators. Before selecting the data of indicators, the applicability and rationality of indicators should be studied. Therefore, the selection of competitiveness evaluation indicators of B2B e-commerce companies must be based on exact standards. The selection principles of indicators in this study are listed as follows.

1. Systematic principle: there are many and complex indicators affecting the competitiveness of B2B e-commerce companies. Considering that B2B e-commerce companies have many business activity procedures and many elements that play a role in all links of activities, the competitiveness evaluation indicators of B2B e-commerce companies must be determined from the perspective of the overall system [15].
2. Scientific principle: the scientific principle has corresponding restrictions on the number, level, and contribution of indicators, and the number of indicators should not be too much or too little. If there are too many indicators, the level of the subcategory is too small, and the evaluation system focuses too much on the details of the competitiveness of B2B e-commerce companies, so it is impossible to study and evaluate the competitiveness of B2B e-commerce companies from a comprehensive perspective, which often makes the contents overlap and the indicators can be replaced with each other. The small number of indicators is not conducive to a detailed and better reflection of the competitiveness of B2B e-commerce enterprises. Each evaluation index has its own significance and scope of action, so the principle of scientificity must be followed [6].
3. Effectiveness principle: when screening the competitiveness evaluation indicators of B2B e-commerce companies, the index data should be available and easy to collect. In addition, the data should not be redundant. The evaluation index system should be improved to the greatest extent, and the value of specific indicators can be run, tested, and verified in the selected method and model software.

### 3.2. Selection of Evaluation Methods for B2B e-Commerce Platform Enterprise Competitiveness

There are many evaluation methods for the competitiveness of B2B e-commerce enterprises [16]. Due to the two sides of things, each evaluation method also has two sides of advantages and disadvantages. Based on the industry characteristics and the specific development of enterprises, it is very important to adopt appropriate methods [17]. This paper summarizes some common evaluation methods of e-commerce enterprise competitiveness, which are discussed as follows.

1. *Principal Component Analysis*
2. The first principal component explains the largest variance, and each secondary component is limited by orthogonality with the previous component. Generally speaking, the first few principal components can explain most of the variance of the original data set [18]. In evaluating the competitiveness of e-commerce enterprises, principal component analysis is mostly applied to the eigenvector decomposition and implementation of correlation matrix [19]. The high-dimensional data set cannot be represented by graphics, and the principal component analysis method can identify the index correlation and patterns in the high-dimensional data set.
3. *Fuzzy Comprehensive Evaluation Method*
4. When making a comprehensive judgment or decision on something, it is a combination of qualitative and quantitative methods to solve the fuzzy information that cannot be solved by other methods [20]. Fuzzy evaluation method can not only sort and evaluate the research object according to the comprehensive score, but also divide it into different grades. Evaluating the competitiveness of B2B e-commerce enterprises is a complex evaluation process with multiple factors and indicators. It cannot be simply divided into “good” or “poor” [21]. When evaluating the competitiveness of B2B e-commerce enterprises, most scholars adopt the decision analysis method based on fuzzy consistency theory. The main feature of fuzzy comprehensive evaluation method is that it can reasonably manage the initiative and fuzziness of human thinking so as to overcome the problem of single result of traditional mathematical methods.
5. *Grey Relational Evaluation Method*
6. In grey system, some information is clear, but others are not. Grey correlation is the variability of the relationship between things or the variability of the relationship between system factors and main activity factors. Grey correlation analysis is one of the important contents of grey system theory research. Its basis is the similarity or difference between the main development trend factors to measure the proximity between these elements [22, 23].

Through the summary of the above B2B e-commerce enterprise competitiveness evaluation methods, it can be seen that these evaluation theories have their own advantages, but the disadvantages are also obvious [24]. Some are too subjective, some do not have comparative function, and some fail to accurately and reasonably evaluate the competitiveness of complete B2B e-commerce enterprises. At the same time, B2B e-commerce enterprise competitiveness evaluation refers to the factors closely related to the enterprise's scale, operation ability, viability, growth ability, technical ability, and so on. It is worth noting that various indicators have nonlinear correlation with each other [25].

### 3.3. Design of B2B e-Commerce Enterprise Competitiveness Evaluation Model Based on BP Neural Network

Improving the number of hidden layers of neural network can improve the nonlinear mapping of neural network, and the number of hidden layers should not be as many as possible. When the number of hidden layers is higher than the specified value, the performance of hidden layer will be weakened. Generally speaking, three-layer BP neural network can perform nonlinear mapping from *n*-dimension to *m*-dimension in any case.

#### 3.3.1. Enter the Number of Layer Nodes

The number of input layer nodes is consistent with the number of parameters presented to the network as input. According to the B2B e-commerce enterprise competitiveness evaluation index system established above, the number of secondary indicators is the number of nodes in the input layer, which is 16.

#### 3.3.2. Number of Output Layer Nodes

Because the research on the competitiveness of B2B e-commerce enterprises finally needs to calculate its competitiveness output value, there is only one value in the output layer, and the number of nodes in the output layer is 1.

#### 3.3.3. Number of Hidden Layer Nodes

In order to obtain efficient, accurate, and reasonable results in a limited time, it is very necessary to determine a reasonable number of hidden layer nodes. There is no general and suitable method to determine the number of neurons in the hidden layer. The following three expressions can be selected as a reference:

(1) $$\begin{array}{c} \sum_{i=0}^{n}C_{M}^{i}>k,\\ M=\sqrt{n+m}+a,\\ M=\log_{2}n, \end{array}$$

where *M* is the number of neurons in the hidden layer, *k* is the number of samples, and *a* is a constant between [0, 10], and *m* and *N* are the number of neurons in the output layer and input layer, respectively.

#### 3.3.4. Activation Function

Generally speaking, BP neural network often uses linear function (purelin) and nonlinear sigmoid function (*S*-type function). *S*-type function includes logarithmic function and tangent function. As shown in formulas (2) and (3), its value range is in the range of [0, 1] and [−1, 1], respectively.

(2) $$\begin{array}{c} \varphi \left(x\right)=\frac{1}{1+e^{-x}}, \end{array}$$

(3) $$\begin{array}{c} \varphi \left(X\right)=\frac{e^{x}-E^{-x}}{e^{x}+e^{-x}}. \end{array}$$

When dealing with nonlinear problems, in order to ensure the range of output values, nonlinear functions are usually used from input layer to hidden layer, and linear functions are used from hidden layer to output layer. After data standardization, the input layer meets the value range requirements of logarithmic sigmoidal function mapping within [0, 1]. Therefore, the function from input layer to hidden layer selected in this paper is logarithmic sigmoidal function, and the function from hidden layer to output layer uses purelin function. The operation process of the activation function is as follows:

For the *s*th data, the input of the *j*th hidden neuron is

(4) $$\begin{array}{c} {\text{net}}_{ij}^{s}=\sum_{i=1}^{16}w_{ij}I_{t}^{s}. \end{array}$$

The corresponding outputs are

(5) $$\begin{array}{c} h_{j}^{s}=\varphi \left({\text{net}}_{j}^{s}\right),\\ =\varphi \left(\sum_{i=1}^{16}w_{ij}I_{i}^{s}\right). \end{array}$$

Therefore, the input of the *k*th output unit is

(6) $$\begin{array}{c} Q_{k}^{s}=\varphi \left({\text{net}}_{k}^{s}\right),\\ =\varphi \left(\sum_{j=1}^{14}{\bar{w}}_{jk}h_{j}^{s}\right),\\ =\varphi \left(\sum_{j=1}^{14}{\bar{w}}_{jk}\varphi \left(\sum_{i=1}^{16}w_{ij}I_{I}^{s}\right)\right). \end{array}$$

#### 3.3.5. Training Function

Training function is also an important parameter of BP neural network. Each training function corresponds to its own algorithm. The training algorithm needs to be selected according to the specific conditions, such as the research problem itself and training samples. Different training algorithms have different space storage, search mode, number of iterations, amount of calculation, calculation speed, convergence speed, and generalization ability. Select traingdx training function for network training.

### 3.4. BP Neural Network Training Sample Collection

The selection of BP neural network training samples should be reasonable and general, and the data collection should be objective, scientific and respect the facts [26]. Since the data of B2B e-commerce listed companies are open and transparent, the data of B2B e-commerce listed companies selected in this paper are from the 2016 annual report and relevant statistical reports. When selecting B2B e-commerce enterprises, they should be selected in a balanced manner among listed companies at all levels and can represent B2B e-commerce companies at all levels. The number of B2B e-commerce enterprise training samples should be objective and feasible. If the number is too small, it is difficult to ensure the demand for errors, making the evaluation conclusion inaccurate and scientific and unable to properly explain the samples and indicators.

### 3.5. Standardized Processing of Sample Data

This paper collects the relevant data of B2B e-commerce enterprises according to the specific evaluation indicators. In this case, it is necessary to standardize the data to eliminate these obstacles. In this paper, maxmin function is used to standardize the original data, which is transformed into the value between (0, 1), so as to facilitate the training and learning of BP neural network. maxmin function formula is as follows:

(7) $$\begin{array}{c} y_{i}=\frac{x_{i}-x_{\min}}{x_{\max}-x_{\min}}, \end{array}$$

where *x*_*i*_ is the initial data, *x*_min_ and *x*_max_ are the minimum and maximum values of the same index, respectively, and *y*_*i*_ is the result of standardization processing.

## 4. Results and Analysis

### 4.1. BP Neural Network Training

#### 4.1.1. Determine the Expected Value of Network Samples

In general, the expected value of BP neural network is the actual value after quantification. However, the competitiveness of B2B e-commerce enterprises covers a wide range and is complex, and the competitiveness value is not clear. Therefore, the weight of each index in the evaluation index system is calculated by the combined weight method, and then the competitiveness value of B2B e-commerce enterprises is obtained by the weighted summation method with the standardized data. The expected value of BP neural network training sample is the weighted summation value. As for the determination of evaluation index weight, scientific and reasonable methods need to be used. Generally, scholars mostly use subjective methods such as Delphi and analytic hierarchy process, and some scholars use more objective entropy weight method to obtain index weight. The proportion of subjective elements is relatively strong, and the result will produce a considerable degree of bias. Generally, it is difficult to meet the objective evaluation conditions, it is difficult to reflect the preference of raters, and sometimes it may deviate from the wishes of raters. In order to avoid the above problems and calculate a relatively objective and reasonable weight value, the evaluation model in this paper adopts the method of combined weight coefficient; namely,

(8) $$\begin{array}{c} W_{j}=\alpha W_{j}^{s}+\left(1-\alpha \right)W_{j}^{\circ }, \end{array}$$

where *W*_*J*_ is the combined weight coefficient of index *J*, *W*_*J*_^*s*^ is the subjective weight coefficient of index *j*, *W*_*j*_° is the objective weight coefficient of index *j*, *α* is the subjective preference coefficient, and (1 − *α*) is the objective preference coefficient, *α* ∈ [0,1]. The function is established for the purpose of minimizing the sum of squares of deviations between subjective weight, objective weight, and combined weight:

(9) $$\begin{array}{c} \min z=\sum_{j=1}^{m}\left[{\left(W_{J}-W_{J}^{s}\right)}^{2}+{\left(W_{J}-W_{J}^{\circ }\right)}^{2}\right]. \end{array}$$

Find the first derivative of equation (8) and make it 0 to obtain *α*  = 0.5.

#### 4.1.2. Subjective Weight Calculation

*G*1 method is derived from the reference and innovation of analytic hierarchy process, which overcomes the shortcomings of AHP and omits the step of consistency check. In order to keep generality, let *X*_1_, *X*_2_, ∧, *X*_*m*_(*m* > 2) be *m* indexes after ensuring consistency and dimensionlessness. If the importance of index *x* is higher (or not lower) than *x*_*j*_, record *x*_*i*_ = *x*_*j*_. If the importance of index *X*_1_, *X*_2_, ∧, *X*_*m*_(*m* > 2) is *x*_1_^·^ = *x*_2_^·^ = ∧ = *x*_*m*_^·^ compared with an evaluation standard, it indicates that the sequential relationship between indexes *X*_1_, *X*_2_, ∧, *X*_*m*_(*m* > 2) is established according to “ = ”. For the indicator set {*X*_1_, *X*_2_, ∧, *X*_*m*_}, establish sequential connection according to the following process:

In the index set {*X*_1_, *X*_2_, ∧, *X*_*m*_}, select the most important index for an evaluation standard and record it as *X*_1_^*∗*^. Among the remaining *m* − 1 indicators, for a certain evaluation standard, select the most important indicator, which is recorded as *X*_2_^*∗*^. Among the remaining *m* − (*k* − 1) indicators, the most important one for a certain evaluation standard is selected and recorded as *X*_*k*_^*∗*^.

*X*_*J*_^*∗*^ is used to represent the *j*th index (*J* = 1, 2,…, *M*) of {*x*_*j*_} arranged in order relationship, from which a unique-order relationship can be obtained. Then, calculate the importance of adjacent indicators. If the researchers' importance ratio between *x*_*k*−1_ and *x*_*k*_ is *r*_*k*_=*W*_*k*−1_/*W*_*k*_, the relative importance of each indicator can be calculated according to the order relationship between the previous indicators. See Table 1 for the value of *r*_*k*_.

Firstly, this paper calculates the weights *W*_1_, *W*_2_,…, *W*_5_ of five primary indicators: enterprise scale (*x*_1_), enterprise benefit (*x*_2_), enterprise financial ability (*x*_3_), enterprise growth ability (*x*_4_), and enterprise technical ability (*x*_5_). According to Definition 2, the only order relationship between them is *x*_1_^*∗*^ > *x*_2_^*∗*^ > *x*_3_^*∗*^ > *x*_4_^*∗*^ > *x*_5_^*∗*^, and their weights under the order relationship are *W*_1_^*∗*^, *W*_2_^*∗*^,…, *W*_5_^*∗*^.

Then, there are

(10) $$\begin{array}{c} r_{2}=\frac{W_{1}^{*}}{W_{2}^{*}},\\ =1.6,r_{3},\\ =\frac{W_{2}^{*}}{W_{3}^{*}},\\ =1.4,r_{4},\\ =\frac{W_{3}^{*}}{W_{4}^{*}},\\ =1.3,r_{5},\\ =\frac{W_{4}^{*}}{W_{5}^{*}},\\ =1.1. \end{array}$$

Restore the weight of the corresponding indicator according to the corresponding relationship, and get

*W*_1_=*W*_4_^*∗*^=0.1295=*W*_2_=*W*_2_^*∗*^=0.2292, *W*_3_=*W*_5_^*∗*^=0.1145, *W*_4_=*W*_1_^*∗*^=0.3667, *W*_5_=*W*_3_^*∗*^=0.1637. Similarly, the weights of the remaining 16 secondary indicators can be obtained, and the results are shown in Table 2.

Entropy is the quantitative unit of average information in information theory. In information theory, the information quantity of the *i*th signal input in an information channel is recorded as *I*_*l*_, *I*_*l*_=−ln*p*_1_, where *p*_1_ is the occurrence probability of the signal. The increase of information indicates that entropy is decreasing, and entropy can calculate the amount of information. Set *x*_*ij*_(*l*=1,2,…, *n*; *j*=1,2,…, *m*) as the observation data of the *j*th index of the *i*th system. For the known *I* and *j*, the higher the value, the more information the index carries and transmits. The final result of objective weight is shown in Table 3.

#### 4.1.3. Combined Weight Calculation

It can be seen from the above that *α*=0.5 and formula (8) shows that the combined weight *W*_*J*_=0.5*W*_*J*_^*S*^+0.5*W*_*J*_°. The final result is shown in Table 4.

Based on the final combination weight after calculation, the expected value of 23 companies is calculated by weighted summation of the standardized sample data, that is, the competitiveness expected value of the selected 23 B2B e-commerce enterprises. The results are shown in Table 5.

### 4.2. Training and Result Analysis of BP Neural Network

#### 4.2.1. Determine the Number of Hidden Layers and Elements of the Network

In order to obtain efficient, accurate, and reasonable results in a limited time, it is very necessary to determine a reasonable number of hidden layer nodes. At present, there is no scientific and reasonable analysis formula that can be used to solve the correct number of neuron nodes. The general practice is to use the experimental formula to deduce the estimated value;

∑_*l*=0_^*n*^*C*_*M*_^*i*^ > *k*, *K* is the number of samples 23, *M* is the number of neurons in the hidden layer, and *N* is the number of neurons in the input layer 16. If *I* > *m*, specify *C*_*M*_^*i*^=0;

$M=\sqrt{n+m}+a$ , *M* and *N* are the number of neurons in the output layer and input layer, respectively, 1 and 16. *A* is a constant between [0, 10]; then the value range of *M* is [4, 13];

*M*=log_2_*n*, *N* is the number of neurons in the input layer; then *M* is 4.

To sum up, the number of hidden layer nodes *m* is within the range of [4, 13], and the specific value must be trained by BP network for many times, which is determined according to the number of iterations and training accuracy. Take the integer between [4, 13] and set the target accuracy to 1 × 10^–5^; the number of training times is 5000. After repeated experiments, the number of hidden layer elements is finally confirmed as 14.

#### 4.2.2. Training Results

The neural network is trained with the help of the function netainparam in the MATLAB neural network toolbox. The function includes the maximum learning times of parameters, the maximum allowable error, that is, the convergence accuracy target, the minimum allowable time, and so on. The maximum learning times is set to 5000 times. Generally, the smaller the convergence accuracy target is, the more accurate the training of the network can be guaranteed. Set it to a sufficiently small accuracy of 1 × 10^–5^; other parameters are set as default values.

20 B2B e-commerce enterprises are randomly selected as training samples to train the neural network. When the training times reach 3297 times, the sample mean square error is 9.9869*e* − 06, and the training network converges. The results are shown in Figure 2.

Then, the trained neural network is tested by using the samples of business Bao *A*3, agricultural products *A*12, and Baoxin software *A*19. The data of the three test samples are input into the trained BP neural network, and the output results are 0.1531, 0.1371, and 0.1557, respectively (Table 6).

According to Table 6, the maximum absolute error between the output value of the test sample and the expected value is less than 0.007, and the maximum relative error is less than 0.05. The error results of the test and the training sample are very close. The established BP neural network has good performance and can be used to evaluate the competitiveness of B2B e-commerce companies. According to the training results of BP neural network, the competitiveness ranking of B2B e-commerce enterprises is obtained, as shown in Table 7.

By ranking the competitiveness of B2B e-commerce by BP neural network, we can understand the competitiveness of B2B e-commerce in China. The competitiveness of B2B e-commerce enterprises in various fields reflects the growth of different companies. This paper analyzes these 23 companies with the method of classification research. First, Figure 3 shows the competitiveness of these 23 companies.

Through the comparison between Zhongyeda and Hikvision, as shown in Figure 4, Hikvision is the only e-commerce concept enterprise focusing on the Internet of things and related businesses. The enterprise has a large volume and has invested a lot of energy in R & D personnel and R & D investment. Under the favorable economic and policy background of the Internet of things industry, its total sales, in the leading position of these 23 enterprises. Zhongyeda is mainly engaged in the distribution of industrial electrical products. The company has established an industrial electrical distribution network, which belongs to a professional vertical e-commerce. Its ranking is lower because the enterprise scale is relatively small, the enterprise profitability is poor, and it does not pay much attention to R&D.

Among the 23 B2B e-commerce enterprises selected in this paper, state-owned holding enterprises include Hikvision, small-commodity city, Longping Hi-Tech, and Haihong Holdings. As shown in Figure 5, these state-owned holding enterprises are relatively competitive, mainly in terms of enterprise scale, operating income and profit, brand value, and R & D investment. On the one hand, state-owned holding enterprises have many assets and large enterprise volume, which occupy natural advantages in capital and policies. On the other hand, state-owned holding enterprises pay more attention to comprehensive development, so they will invest capital and technology in the improvement and cultivation of each factor, which also improves their comprehensive competitiveness overall. In contrast, the turnover rate of fixed assets of state-owned holding enterprises is relatively small, the utilization efficiency of fixed assets is weak, and the asset utilization degree of enterprises is low, which limits the profit potential of the company to a certain extent.

Platform e-commerce mainly includes Focus Technology, Shanghai Steel Union, Business treasure, Commodity city, Zhejiang Oriental, Ruimaotong, Tengbang International, Oriental Group, and so on. Platform e-commerce shows bipolar development, with small-commodity city, Oriental Group, Ruimaotong, and Focus Technology ranking in the top ten, as shown in Figure 6. These companies are outstanding in brand value, technological innovation, and asset operation, so they rank high. Because enterprises pay more attention to the construction of e-commerce platform, they start early and involve deep industrial fields. After a long time of capital, talents, and brand precipitation, they have formed unique competitiveness in the field of comprehensive platform and have a high market share. As these platforms involve a relatively wide range of industrial fields, their overall financial capacity is not comparable to that of state-owned enterprises.

As shown in Figure 7, the platform e-commerce of Business treasure, Smart energy, Zhejiang Oriental, and Zhongyeda rank lower in 17, 19, 21, and 23, respectively, so their competitiveness is relatively weak because they are relatively backward in terms of enterprise scale, profitability, capital operation, and innovation ability.

E-commerce service enterprises mainly include Wangsu Technology, Altega, Baoxin software, and Zhejiang University Wangxin, ranking 2, 11, 15, and 22, respectively, as shown in Figure 8. Although the scale of these four enterprises is roughly the same, Wangsu technology has a relatively large competitive advantage in enterprise efficiency, financial ability, growth ability, and technical ability, mainly due to its preference for technological development and technological innovation. Enterprise users have included various websites, online game enterprises, and operators, which has brought relatively high profitability.

### 4.3. Improving Enterprise Competitiveness and Innovation

According to the analysis and summary of the competitiveness of the above enterprises, corresponding improvement suggestions should be put forward according to the actual situation of various enterprises. The efficiency of state-owned holding enterprises in the utilization of fixed assets is relatively low, and the asset utilization degree of enterprises is low. The enterprise shall formulate the use plan of fixed assets, analyze the demand for fixed assets, complete the strategic option analysis, list the asset items, formulate the management performance measures and asset management plan, complete the capital budget, and finally implement it with the approval of the management. In addition, the company should also pay attention to the acquisition of fixed assets. The goal is to enable the enterprise to obtain reasonable and useful property for the enterprise in the most economical and effective way. The acquisition solves the problem of initial control of assets. The more common ways are purchase, value exchange, accepting government or individual donations, tax foreclosure, and so on. Implement the operation and maintenance of fixed assets in accordance with the maintenance strategies and policies under the framework of laws and regulations. In addition, enterprises should change their management concept from extensive to intensive, strengthen the level of asset management, and focus on internal asset management. In addition, we should scientifically adjust the enterprise asset structure and combine the assets with relatively low risk in order to seek the maximum benefits.

The competitiveness level of platform e-commerce is characterized by polarization. For backward companies, because they are relatively backward in company scale, profitability, capital operation, or innovation ability, they should clarify their business areas and strive to seek inter industry cooperation. In particular, these enterprises should pay attention to the application of business intelligence and collect and convert the internal and external resources of the enterprise from multiple angles into a structured data system so as to shorten the time to obtain relevant information and realize the efficient utilization of resources. It is better for enterprises to introduce REP system to realize the efficient management and operation of sales, marketing, manufacturing, operation, logistics, procurement, finance, new product development, and human resources and provide the basis for effective e-commerce. Specifically, it controls and confirms the company's cash flow in real time, promotes the implementation of interdepartmental cooperation, and reduces the time required to generate regular reports. Through transaction data analysis and prediction of business trends, improve profitability, enable financial personnel to quickly create financial revenue reports and expenses, improve relationship management with suppliers, facilitate efficient management of employees, and provide online access to data so as to save access time and other aspects. For the top platform e-commerce enterprises, their financial ability is relatively weak, which may hinder the effective investment of enterprises and affect the ability of enterprises to further grow. Enterprise financial ability is reflected in the realization of organizational objectives and production efficiency. The higher the financial ability, the lower the cost and the improvement of enterprise value. On the one hand, enterprises should pay attention to internal financing, which refers to the funds independently obtained by enterprises, mainly including retained earnings and depreciation. This is not only the key element of the company's survival and development, but also an effective way to improve the competitiveness of e-commerce enterprises in finance. On the other hand, the company should also pay attention to the integration of external financial resources because this is the key factor for the rapid growth and competitiveness of the company. In addition, the effective use of resources, effective control, effective management of working capital, and reliable financial prediction are very important to the improvement of enterprise financial ability.

## 5. Conclusion

This paper innovates the business evaluation system based on BP neural network and artificial intelligence technology. Taking 23 listed B2B e-commerce enterprises as analysis samples, this paper evaluates the competitiveness of B2B e-commerce enterprises with specific indicators such as total assets, total employees, total sales, proportion of R & D personnel, and proportion of R & D investment in total sales. The neural network is trained and tested with the data of 23 enterprises. Finally, the trained network is used to obtain the competitiveness value of B2B e-commerce enterprises, analyze the evaluation results, point out the advantages and disadvantages for different types of enterprises, and provide relevant improvement suggestions. This paper selects 23 B2B e-commerce enterprises and compares the competitiveness gap between enterprises horizontally. For a specific enterprise, it does not collect, sort out, and analyze the company data for many consecutive years, ignoring the vertical analysis and exploration of the company's competitiveness. Therefore, the follow-up research work should take a representative B2B e-commerce enterprise as the research object, study the development route of its competitiveness, study and analyze the reasons for the enhancement or weakening of enterprise competitiveness, and provide experience and reference for relevant enterprises in B2B e-commerce industry.

## Figures and Tables

**Figure 1:** Business model innovation process integration model.

**Figure 2:** Convergence accuracy of BP neural network training results.

**Figure 3:** Evaluation results of B2B e-commerce enterprise competitiveness based on BP neural network.

**Figure 4:** Comparison of evaluation index values between Zhongyeda and Hikvision.

**Figure 5:** Competitiveness factors of state-owned holding enterprises.

**Figure 6:** Competitiveness factors of top ten platform e-commerce enterprises.

**Figure 7:** Competitiveness factors of platform e-commerce enterprises ranked lower.

**Figure 8:** Competitiveness factors of e-commerce service enterprises.

**Table 1:** *r*_*k*_ value reference table.

*r*_*k*_	Value reference
1.0	Indicators *x*_*K*−1_ and *x*_*K*_ are of the same importance
1.1	The ratio of indicators *x*_*K*−1_ and *x*_*K*_ is between equally important and slightly important
1.2	Indicator *x*_*K*−1_ is slightly more important than *x*_*K*_
1.3	The ratio of index *x*_*K*−1_ to *x*_*K*_ is between slightly important and obviously important
1.4	The index *x*_*K*−1_ is obviously more important than *x*_*K*_
1.5	The ratio of index *x*_*K*−1_ to *x*_*K*_ is between obviously important and strongly important
1.6	Index *x*_*K*−1_ is more important than *x*_*K*_
1.7	The ratio of index *x*_*K*−1_ to *x*_*K*_ is between strongly important and extremely important
1.8	Index *x*_*k*−1_ is more important than *x*_*k*_

**Table 2:** Subjective weight of indicators.

Primary index	Secondary index	Secondary index weight
Enterprise scale	Total assets *X*1	0.0396
	Total number of employees *X*2	0.0305
	Total sales *X*3	00594
Enterprise benefit	Operating net profit margin *X*4	0.0440
	Return on total *X*5	0.0572
	Return on net *X*6	0 0366
	Year on year growth rate of total operating revenue *X*7	00915
Enterprise financial capability	Current ratio *X*8	0.0496
	Quick ratio *X*9	0.0354
	Asset liability ratio *X*10	00295
Enterprise growth ability	Fixed assets turnover *X*11	0.0711
	Growth rate of total assets *X*12	0.0646
	Net interest rate of total assets *X*13	0.0924
	Brand value *X*14	0.1386
Enterprise technical capability	Proportion of R & D personnel *X*15	0.0744
	Proportion of R & D investment in total sales *X*16	0.0893

**Table 3:** Objective weight of indicators.

Primary index	Secondary index	Secondary index weight
Enterprise scale	Total assets *X*1	0.0403
	Total number of employees *X*2	0.0477
	Total sales *X*3	0.0593
Enterprise benefit	Operating net profit margin *X*4	0.0301
	Return on total assets *X*5	0.0347
	Return on net assets *X*6	0.0212
	Year-over-year growth rate of total operating revenue *X*7	0.0804
Enterprise financial capability	Current ratio *X*8	0.0371
	Quick ratio *X*9	0.0490
	Asset liability ratio *X*10	0.0139
Enterprise growth ability	Fixed assets turnover *X*11	0.1799
	Growth rate of total assets *X*12	0.0897
	Net interest rate of total assets *X*13	0.0365
	Brand value *X*14	0.0916
Enterprise technical capability	Proportion of R & D personnel *X*15	0.0710
	Proportion of R & D investment in total sales *X*16	0.1176

**Table 4:** Combination weight table.

Primary index	Secondary index	Secondary index weight
Enterprise scale	Total assets *X*1	0.0400
	Total number of employees *X*2	0.0389
	Total sales *X*3	0.0594
Enterprise benefit	Operating net profit margin *X*4	0.0370
	Return on total *X*5	0.0459
	Return on net *X*6	0.0289
	Year on year growth rate of total operating revenue *X*7	0.0859
Enterprise financial capability	Current ratio *X*8	0.0433
	Quick ratio *X*9	0.0422
	Asset liability ratio *X*10	0.0217
Enterprise growth ability	Fixed assets turnover *X*11	0.1255
	Growth rate of total assets *X*12	0.0772
	Net interest rate of total assets *X*13	0.0644
	Brand value *X*14	0.1151
Enterprise technical capability	Proportion of R & D personnel *X*15	0.0727
	Proportion of R & D investment in total sales *X*16	0.1034

**Table 5:** Expected values of 23 samples.

Enterprise	Expected value
Focus technology *A*1	0.203585113
Shanghai steel union *A*2	0.207850128
Business treasure *A*3	0.153025267
Small-commodity city *A*4	0.247207125
Zhejiang Dongfang *A*5	0.120882515
Hikvision *A*6	0.439256148
Smart energy *A*7	0.127821756
Zhongyeda *A*8	0.101404129
Ruimaotong *A*9	0.318937614
Tengbang International *A*10	0.153135323
Zheshang Zhongtuo *a*11	0.16045568
Agricultural products *A*12	0.13641545
Deep SEG *A*13	0.159326222
Longping Hi-Tech *A*14	0.20954871
Oriental group *A*15	0.246449142
Wangsu Technology *A*16	0.424062233
Altega *A*17	0.189879302
Zdg new *A*18	0.109041243
Baoxin software *A*19	0.155111216
Changjiang investment *A*20	0.125483542
Sinotrans Development *A*21	0.175951754
Haihong Holdings *A*22	0.293397612
Shenzhen Huaqiang *A*23	0.196212136

**Table 6:** Comparison of test sample output results and expected values.

B2B e-commerce enterprise	Network output value	Expected value	Absolute error	Relative error
Business treasure *A*3	0.1531	0.1530	0.0001	0.0007
Agricultural products *A*12	0.1371	0.1364	0.0007	0.0051
Baoxin software *A*19	0.1557	0.1551	0.0006	0.0039

**Table 7:** Competitiveness ranking of B2B e-commerce enterprises.

Enterprise	Competitive power	Ranking
Focus technology *A*1	0.2035	9
Shanghai steel union *A*2	0.2080	8
Business treasure *A*3	0.1513	17
Small-commodity city *A*4	0.2462	5
Zhejiang Dongfang *A*5	0.1216	21
Hikvision *A*6	0.4383	1
Smart energy *A*7	0.1264	19
Zhongyeda *A*8	0.1012	23
Ruimaotong *A*9	0.3179	3
Tengbang International *A*10	0.1540	16
Zheshang Zhongtuo *A*11	0.1577	13
Agricultural products *A*12	0.1353	18
Deep SEG *A*13	0.1610	14
Longping Hi-Tech *A*14	0.2053	7
Oriental Group *A*15	0.2466	6
Wangsu Technology *A*16	0.4232	2
Altega *A*17	0.1910	11
ZDG new *A*18	0.1113	22
Baoxin software *A*19	0.1530	15
Changjiang Investment *A*20	0.1236	20
Sinotrans Development *A*21	0.1761	12
Haihong Holdings *A*22	0.2956	4
Shenzhen Huaqiang *A*23	0.1953	10

## Data Availability

No data were used to support this study.
